This article has been retracted.

# Acute Thrombolytic Therapy Combined with the Green Channel Can Reduce the Thrombolytic Time and Improve Neurological Function in Acute Stroke Patients

**DOI:** 10.1155/2022/1127159

**Published:** 2022-06-27

**Authors:** Zhen Hong, Mingming Zheng, Yan Li, Shaoquan Li, Qingran Liu, Songwang Xie, Junyong Wang, Jian Wang, Yongchang Liu

**Affiliations:** Department of Neurovascular Intervention, Cangzhou Central Hospital, Cangzhou, Hebei, China

## Abstract

**Objective:**

To explore the effect of acute thrombolytic therapy combined with the green channel on the thrombolytic time and neurological function in acute stroke patients.

**Methods:**

A total of 100 acute stroke patients admitted to our hospital from August 2016 to August 2019 were recruited as the research cohort. In experimental group, 50 patients were administered green channel combined with acute thrombolytic therapy, while the patients in control group were administered general therapy. The thrombolytic times, the muscle strength grades, the FMA scores, the Barthel index levels, the NIHSS and SSS scores, the SAS and SDS scores, the arterial pressure and heart rates, the total effective rates, the incidences of postoperative adverse reactions, and the satisfaction levels were compared between the two groups.

**Results:**

The thrombolysis times in experimental group were shorter than those in control group. In experimental group, there were more patients with muscle strength grades 4 and 5 (*P* < 0.05), the FMA and Barthel index levels were higher, the NIHSS and SSS (*P* < 0.05) and the SAS and SDS scores were lower, the arterial pressure and heart rates were lower (*P* < 0.05), the incidence of postoperative adverse reactions was lower (*P* < 0.05), the total efficiency was higher (*P* < 0.05), and the satisfaction level was higher (*P* < 0.05).

**Conclusion:**

Acute thrombolytic therapy combined with the green channel can significantly reduce the thrombolytic time and improve the neurological function in acute stroke patients.

## 1. Introduction

Acute stroke due to cerebral infarction is a very common disease, especially in the middle-aged and elderly population, with a poor prognosis and high mortality rate that will have a significant impact on daily life [1–4]. In serious cases, the normal exercise of patients will be impaired, eventually even leading to disability [5, 6]. As a result of the development of atherosclerosis, intracranial blood vessels become embolised, in most cases blocking the flow of blood to a part of the brain, leading to massive cerebral infarction and stroke [7, 8]. Thrombolysis has always been a therapeutic method for stroke caused by obstruction [9]. Intravenous thrombolytic therapy can rapidly restore cerebral blood flow, can improve brain tissue metabolism, can protect the ischaemic semidark zone tissue around the infarct with only functional changes from forming necrosis, can maximise the signs and symptoms of neurological deficits, and can reduce the mortality and disability of patients [10]. Urokinase, an enzyme that acts directly on the endogenous fibrinolytic system, is derived from the urine of healthy individuals and has been widely used to treat thrombolysis in stroke patients [11]. It catalyses the conversion of a fibrin hydrolase, plasminogen, into an active form of plasmin and plays a thrombolytic role [12]. A variety of clinical studies on stroke are also treated with urokinase activating fibre enzymic, which is a kind of acute thrombolytic therapy [13, 14].

Untreated cerebral ischaemia in stroke patients has the potential to cause cognitive impairment, which not only has a serious impact on social functioning but also places a burden on family care [15]. There is also a risk of motor dysfunction, most commonly resulting in hemiparesis and, in severe cases, bed rest [16]. If the ischaemic stroke is large, it may even cause the patient to become unconscious and endanger his or her life. In the acute phase, ischaemic stroke can also lead to complications, such as lung infection, stress ulcers, and deep vein thrombosis of the lower limbs [17]. The urgency of acute stroke treatment has led to the creation of a green channel for patients in many clinical settings so that they can receive timely and effective treatment [18, 19]. In recent years, there have been many studies on the effects of green channel and thrombolytic therapy, but there are few studies that evaluate the effects of green channel and thrombolytic therapy based on mental health status, nerve function, limb function, and other indicators.

This study aimed to analyse the effect of acute thrombolytic therapy combined with the green channel on patients with acute stroke through their anxiety and depression scores, thrombolytic times, neurological function, and other indicators.

## 2. Materials and Methods

### 2.1. Baseline Data

100 patients with acute cerebral stroke according to Chinese Guidelines for Diagnosis and Treatment of Acute Ischemic Stroke (2014) who were admitted to our hospital from August 2016 to August 2019 were recruited for prospective study and divided into two groups by random number table method, of which 50 patients received green channel combined with acute thrombolysis (experimental group), and 50 cases were given traditional treatment (control group).

#### 2.1.1. Inclusion Criteria

1. Patients with a strong compliance
2. Patients who could correctly understand the instructions of the medical staff during the treatment
3. Patients who could accurately express physical discomfort, patients whose symptoms were stable within the last month, and in whom no new strokes occurred
4. Patients and their families who agreed to the study and who signed the consent form

#### 2.1.2. Exclusion Criteria

1. Patients who suffered from other serious underlying diseases, such as dysfunction of the heart, liver, kidneys, and other internal organs
2. Patients who suffered from mental disorders, such as frequent anxiety, depression, and suicide

This study was approved by our hospitals' ethics committees.

### 2.2. Methods of Treatment

*Experimental Group*. The patient received acute thrombolytic therapy combined with green channel treatment. When the patient is admitted to the hospital, the medical staff needs to make an initial assessment of the patient's vital signs as well as other indicators (muscle tension, state of consciousness, facial expression, etc.) and immediately notify the emergency department. Several departments such as the emergency department, radiology, neurology, and laboratory then need to join forces to set up the green channel immediately. Next, the designated application form was used to avoid having the patient's queue for treatment. At the same time, the attending physician in the department of neurology had to be in place within 5 minutes. The NIHSS (neurological impairment) score scale test and a physical examination were carried out within 10 min [20]. The emergency nurses needed to establish venous channels for the patients within 5 minutes, and they took blood samples and sent them to the department of laboratory for testing. The medical staff in the department of laboratory conducted the blood test within 40 minutes and sent the test results to the corresponding departments. The radiology medical staff performed a brain CT or an MRI examination on the patient within 30 minutes and sent the examination results to the corresponding department. The patient's condition was then assessed by the attending neurologist. With the consent of the patient and family, intravenous thrombolytic therapy with urokinase was performed. Recombinant human tissue fibrinogen activator (rt-PA) was used for thrombolysis. A microcatheter was delivered to the stenosis or occlusion site (the head end was as close to the thrombus as possible) by superselection. The r-tpA (20–30 mg) (average 25 mg) +50 ml normal saline was infused for 30–60 min. The cerebral angiography was reviewed to determine the recanalization of the occluded vessels. After the surgery, heparin was used for 24 hours to maintain normal coagulation function, and the coagulation mechanism was monitored. During the treatment, the thrombolysis was stopped immediately in the case of cerebral haemorrhage, and fresh frozen plasma and platelets were used to maintain fibrin at more than 1 g/L. At the same time, 30 mg of edaravone (Lijun Pharmaceutical Co., Ltd., batch no.: H20120042) was given via intravenous drip twice a day. After 24 h, the skull was reexamined with CT or MRI to confirm that there was no intracranial haemorrhage, and then low-molecular-weight heparin and aspirin were used for anticoagulation. Rehabilitation training was carried out after the operation.

*Control Group*. The patients underwent general therapy [21]. The medical staff needed to diagnose the specific conditions of the patient's disease; then, they formulated a thrombolytic therapy and cooperated with postoperative rehabilitation training.

### 2.3. The Index Levels

#### 2.3.1. Thrombolytic times

The patients' thrombolytic times were observed and compared in the two groups.

#### 2.3.2. Muscle Strength Grades

The patients' muscle strength after the treatment was used as an index to judge the limb recovery levels. Grade 0: The patient cannot feel muscle contractions. Grade 1: The patient had no significant movement, but muscle contractions were possible. Grade 2: The patients was unable to overcome the limb weight movement and the horizontal surface of the movement without load. Grade 3: The patient could move aginst the body's own weight. Grade 4: The patient could exercise to overcome moderate resistance. Grade 5: The patient could move on his or her own.

#### 2.3.3. Limb Function

Before and after treatment for one month, the limb function (FMA) scores [22] and the Barthel index [23] levels were compared to evaluate the patients' limb recoveries. The higher the score, the better the recovery of the limb effect.

#### 2.3.4. Neurological Function and Mental Health

The NIHSS and neurological function scores (SSS) were used to evaluate the neurological function recovery of the patients in the two groups. The better the recovery of a patient's neurological function, the lower the score. The self-rating anxiety scale (SAS) [24] and the self-rating depression scale (SDS) [25] were used to evaluate the mental health levels (20 items, 0–100 points) of the patients in experimental group and control group before the treatment and after the treatment for 1 month. The worse the mental health level of patients, the higher the score.

#### 2.3.5. Arterial Pressure and Heart Rate

After the hospitalization, the patients' arterial pressure and heart rates were measured in real time in the two groups. The patients' arterial pressure and heart rates were compared in the two groups before the treatment and after the treatment for 14 days.

#### 2.3.6. Postoperative Complications

After the operation and for 28 days, the patients' adverse reaction indexes (epilepsy, urinary incontinence, pulmonary infection, and dementia after stroke) were determined and compared.

#### 2.3.7. Total Effective Rate

Criterion of the therapeutic effect: The neurological function improvement rate was over 46%, and the daily living abilities were basically restored (markedly effective). The nerve function improvement rate was 18%∼45%, and the daily living abilities were recovered to a certain extent (effective). The neurological function improvement rate was less than 18%, and the daily living abilities were not restored (ineffective). Total effective rate = markedly effective rate + effective rate.

#### 2.3.8. The Treatment Satisfaction Was Compared in the Two Groups

The treatment satisfaction questionnaire was used to test the patients' satisfaction with treatment. Then, the treatment satisfaction scores of the patients were compared in the two groups. We drew up the test content and evaluation criteria. The total possible score was 100 points, of which 100–85 points was considered satisfactory, more than 70 points was considered basically satisfactory, and less than 70 points was considered unsatisfactory.

### 2.4. Statistical Methods

SPSS 19.0 (AsiaAnalytics, formerly SPSS China) was used for the statistical analysis of the comprehensive data. *X*^2^ tests were used for the count data, such as the baseline data (gender, hypertension or not, hyperlipidaemia, diabetes, incidence of adverse reactions, and total effective rate). The measurement data were expressed as (*X* ± *S*) and *t* tests were used, such as comparing the scores in experimental group and control group. A difference was considered statistically significant when *P* < 0.05.

## 3. Results

### 3.1. Baseline Data of the Patients in Both Groups

There were no significant differences in terms of the baseline data, including gender, age, BMI, smoking history, drinking history, and the obesity status between the two groups (*P* > 0.05) (Table 1).

### 3.2. Thrombolytic Times of the Patients in Both Groups

The thrombolytic time of experimental group was (68.74 ± 10.75), and the thrombolytic time of control group was (145.65 ± 17.45). The thrombolytic time in experimental group was significantly shorter than the thrombolytic time in control group (*P* < 0.05) (Figure 1).

### 3.3. The Muscle Strength Grades of the Patients in Both Groups

There were significantly fewer patients in experimental group with grades 0–3 than there were in control group, and there were significantly more patients in experimental group with grades 4-5 than there were in control group (*P* < 0.05) (Table 2).

### 3.4. Limb Function of Patients in Both Groups

In experimental group, the FMA score was (49.78 ± 4.54) before the treatment and (90.34 ± 7.67) at one month after the treatment. In control group, the FMA score was (49.89 ± 4.68) before the treatment and (79.25 ± 6.23) at one month after the treatment. The FMA score improved in both groups at one month after the treatment, and the FMA score in experimental group was significantly higher than that in control group at one month after the treatment (*P* < 0.05). In experimental group, the Barthel index was (42.89 ± 3.45) before the treatment and (84.65 ± 5.81) at one month after the treatment. In control group, the Barthel index was (43.13 ± 3.24) before the treatment and (74.31 ± 4.45) at one month after the treatment. The Barthel index improved in both groups at one month after the treatment, and the Barthel index in experimental group was significantly higher than it was in control group at one month after the treatment (*P* < 0.05) (Figure 2).

### 3.5. The Neurological Function and Mental Health of the Patients in the Two Groups

#### 3.5.1. Neurological Function

In experimental group, the patients' NIHSS scores were (68.32 ± 5.66) before the treatment and (33.34 ± 2.77) at one month after the treatment. In control group, the patients' NIHSS scores were (68.95 ± 5.87) before the treatment and (46.67 ± 6.23) at one month after the treatment. The NIHSS scores decreased in both groups at one month after the treatment, and the NIHSS scores in experimental group were significantly lower than they were in control group at one month after the treatment (*P* < 0.05). In experimental group, the patients' SSS scores were (24.87 ± 2.42) before the treatment and (12.45 ± 1.31) at one month after the treatment. In control group, the patients' SSS scores were (24.34 ± 2.04) before the treatment and (20.13 ± 0.98) at one month after the treatment. The SSS scores decreased in both groups at one month after the treatment, and the SSS scores in experimental group were significantly lower than they were in control group at one month after the treatment (*P* < 0.05) (Figure 3).

#### 3.5.2. Mental Health

Before the treatment and at one month after the treatment, the SAS scores were (63.87 ± 9.61) and (40.43 ± 5.53), respectively, in experimental group. Before the treatment and at one month after the treatment, the SAS scores were (64.18 ± 9.45) and (52.21 ± 5.43), respectively, in control group. At one month after the treatment, the SAS scores in experimental group were significantly lower than they were in control group (*P* < 0.05). Before the treatment and at one month after the treatment, the SDS scores were (61.13 ± 8.54) and (41.34 ± 5.34), respectively, in experimental group. Before the treatment and at one month after the treatment, the SDS scores were (60.87 ± 8.05) and (53.54 ± 6.45), respectively, in control group. At one month after the treatment, the SDS scores in experimental group were significantly lower than they were in control group (*P* < 0.05) (Figure 4).

### 3.6. Arterial Pressure and Heart Rate in the Two Groups

Before and at one month after the treatment, the arterial pressure in experimental group was (118.12 ± 4.92) mmHg and (96.12 ± 2.02) kPa, respectively. Before and at one month after the treatment, the heart rate in experimental group was (105.88 ± 4.79) bpm and (87.54 ± 3.67) bpm, respectively. Before and at one month after the treatment, the arterial pressure in control group was (117.85 ± 5.28) mmHg and (103.78 ± 3.01) kPa, respectively. Before and at one month after the treatment, the heart rate in control group was (106.24 ± 5.26) bpm and (95.47 ± 3.56) bpm, respectively. The arterial pressure and heart rate were compared between the two groups. The arterial pressure and heart rate in experimental group were significantly higher than they were in control group after the operations (Figure 5).

### 3.7. Postoperative Complications of the Patients in the Two Groups

In experimental group, there was 1 case of epilepsy (2.00%), 1 case of urinary incontinence (2.00%), 1 case of dementia after a stroke (2.00%), and no pulmonary infections, so the incidence of adverse reactions was 6%. In control group, there were 5 cases of epilepsy (10.00%), 5 cases of urinary incontinence (38.00%), 3 cases of pulmonary infection (6.00%), and 2 cases of dementia after a stroke (4.00%), so the incidence of adverse reactions was 30%. The postoperative complication rate in control group was significantly higher than it was in experimental group (*P* < 0.05) (Table 3).

### 3.8. Total Effective Rates of the Patients in the Two Groups

In experimental group, there were 26 cases that were markedly effective, 21 cases that were effective, and 4 cases that were ineffective, for a total effective rate of 92.00%. In control group, there were 18 cases that were markedly effective, 20 cases that were effective, and 12 cases that were ineffective, for a total effective rate of 76%. The total effective rate in experimental group was significantly higher than it was in control group (*P* < 0.05) (Table 4).

### 3.9. Treatment Satisfaction in the Two Groups

In experimental group, there were 35 patients who were satisfied, 14 patients who were basically satisfied, 1 patients who was dissatisfied, for a satisfaction rate of 98.00%. In control group, there were 20 patients who were satisfied, 15 cases who were basically satisfied, and 15 cases who were dissatisfied, for a satisfaction rate of 70.00%. The satisfaction in experimental group was significantly higher than it was in control group (*P* < 0.05) (Table 5).

## 4. Discussion

Cerebral thrombosis is a condition in which the cerebral arteries are thickened, narrowed, or occluded as a result of thrombosis secondary to local vascular disease, resulting in reduced or interrupted blood flow to the brain, ischaemia, hypoxia, necrosis, and focal neurological deficits in brain tissue [26]. As a disease with a high mortality and disability rate, the choice of treatment for acute stroke is undoubtedly very important, and acute thrombolysis is an excellent method of thrombolysis, of which rt-PA is an appropriate choice [27, 28]. In this experiment, the effect of acute thrombolytic therapy combined with the green channel on acute stroke patients was studied. The green life-safety channel for emergency care refers to the principle of prioritising resuscitation, examination, and hospitalization for all patients in critical and serious conditions [29]. When a patient arrives at the hospital, if the onset of stroke is very short, a dedicated person will accompany him to the hospital, examine him, treat him, and give him medication as quickly as possible in order to shorten the delay, because once a stroke occurs, there is a lot of brain cell necrosis, which increases with time [30]. A good green channel for stroke care during this process will allow the patient to be treated as quickly as possible.

Firstly, we compared the thrombolytic times of the patients in the two groups. The results showed that patients receiving green channel and acute thrombolytic therapy had significantly shorter thrombolysis times than those receiving general therapy. rt-PA is a wonderful method for thrombolytic therapy. Its mechanism of action is to catalyse fibrin hydrolase into active fibrinolytic enzymes to achieve a thrombolytic effect. At the same time, rt-PA needs to be completed in a short time; otherwise, the effect will be poor [31]. Meanwhile, acute stroke treatment needs to buy time, so in many cases green channels need to be opened to enable patients to receive timely treatment [32]. In contrast, the patients undergoing the conventional treatment are at a disadvantage. Because the common treatment is not as timely as the acute thrombolysis, the thrombolysis times are significantly shorter than they are in the patients receiving the acute thrombolysis with the green channel. Following this, our results comparing the patients' limb recovery showed that, although all had undergone rehabilitation, patients receiving acute thrombolysis in the green channel generally had muscle strength levels 4 and 5, with higher FMA and BI (i.e., better limb recovery than their counterparts, patients who received general treatment). Based on the timing of previous thrombolysis, patients who underwent acute thrombolysis using the green channel had better thrombolysis results and this group of patients could complete their rehabilitation in a better and more timely manner. As a result, they had better limb recovery.

The patients' neurological function and mental health were also tested in our study. Our study revealed that the SSS and NIHSS scores after the acute thrombolytic therapy using the green channel were lower, and the SAS and SDS scores were also lower. Stroke is caused by cerebral obstruction, which causes ischaemic damage to the brain. Subsequently, inflammatory factors cause vasoconstriction, reduced blood flow, and endothelial cell damage in the brain, resulting in significant impairment of neurological function [33]. During thrombolysis with rt-PA, there is a dynamic balance between coagulation and fibrinolysis, which consumes large amounts of coagulation factors and promotes thrombolysis [34]. Cerebral ischaemic symptoms caused by thrombotic obstruction were correspondingly relieved, with better recovery of brain cells and neurological function. We also compared the overall efficiency, complication rates and patient satisfaction. The results showed that patients treated with acute thrombolysis combined with green channel had a higher overall efficiency and satisfaction rate and fewer complications. According to the results of the thrombolytic times and neurological function recovery, the patients with acute thrombolytic therapy combined with the green channel had shorter thrombolytic times, so their neurological function recovery was better, and their limb function recovery was faster. In addition to lower SDS and SAS scores, we found that their anxiety and depression were better relieved by improvement, resulting in higher overall efficiency and fewer postoperative complications. Therefore, the patients were more satisfied, and the evaluation rate was higher. In the clinical study of Qin et al. on patients with acute cerebral infarction, it was found that green channel and rt-PA thrombolytic therapy had a better effect on thrombus [35]. In the clinical study of intravenous thrombolytic therapy conducted by Liu et al., it was found that reducing the interval time of intravenous thrombolytic therapy in hospital was helpful in accelerating the recovery of patients after stroke [36]. This is similar to this research on the green channel.

Traditional Chinese medicine believes that thrombosis is mostly caused by stagnation of qi and blood, so traditional Chinese medicines for thrombolysis generally have the effect of promoting blood circulation and removing blood stasis [37]. Lysis capsule is mainly composed of Dilong, which has the functions of clearing heat and calming convulsions, promoting blood circulation, and dredging collaterals effect [38]. Xiaoshuan Tongluo capsules can also be used as an auxiliary, which has the effect of promoting blood circulation and removing blood stasis, warming meridians, and dredging collaterals. It is used in the recovery period of meridians and collaterals in stroke caused by qi deficiency and blood stasis and has a certain role in assisting thrombolysis [39]. Chinese herbal medicine Panax notoginseng not only has the effect of promoting blood circulation and removing blood stasis, but also nourishing blood and relieving pain [40]. The anticoagulant effect of Panax notoginseng can increase coronary blood flow, slow down heart rate, control blood pressure, reduce coronary resistance, reduce myocardial oxygen consumption, and prevent platelet aggregation, thereby playing an antithrombotic effect [41].

There are some limitations and shortcomings in this trial. Firstly, this trial only tested partial thrombolysis times and neurological function scores. Secondly, due to equipment limitations, we were unable to explore the target molecules and related pathways that lead to stroke, nor did we perform animal experiments on the related molecules. Hence, in our subsequent studies, we will actively procure equipment to further investigate these molecular mechanisms.

## 5. Conclusion

To sum up, acute thrombolytic therapy combined with the green channel can significantly reduce the thrombolytic times and improve the neurological function in acute stroke patients. It can cure acute stroke patients in a timelier manner, so it is worthy of clinical promotion [42].

## Figures and Tables

**Figure 1:** Comparison of the thrombolytic times in the two groups. The thrombolytic times in experimental group were significantly shorter than they were in control group (*P* < 0.05). *Note*. ^*∗*^ indicates compared with control group, *P* < 0.05.

**Figure 2:** Comparison of the limb function between the two groups. (a) FMA scores in the two groups: The FMA scores of both groups improved at one month after the treatment, and the FMA scores in experimental group were significantly higher than they were in control group at one month after the treatment (*P* < 0.05). (b) Barthel index levels in the two groups: The Barthel index levels improved in both groups at one month after the treatment, and the Barthel index levels in experimental group were significantly higher than they were in control group at one month after the treatment (*P* < 0.05). *Note*. ^*∗*^means a comparison with before the treatment, *P* < 0.05; ^#^means a comparison with control group, *P* < 0.05.

**Figure 3:** Comparison of neurological function between the two groups. (a) NIHSS scores in the two groups: The NIHSS scores were reduced in both groups at one month after the treatment, and the NIHSS scores in experimental group were significantly lower than they were in control group at one month after the treatment (*P* < 0.05). (b) The SSS scores in both groups: The SSS scores decreased in both groups at one month after the treatment, and the SSS scores in experimental group were significantly lower than they were in control group at one month after the treatment (*P* < 0.05). *Note*. ^*∗*^means a comparison with before the treatment, *P* < 0.05; ^#^means a comparison with control group, *P* < 0.05.

**Figure 4:** Comparison of the mental health in the two groups. (a) SAS scores in the two groups: The SAS scores were decreased in the two groups after the treatment, and the SAS scores in experimental group were significantly lower than they were in control group (*P* < 0.05). (b) The SDS scores in the two groups: The SDS scores were decreased in the two groups after the treatment, and the SDS scores in experimental group were significantly lower than they were in control group (*P* < 0.05). *Note*. ^*∗*^means a comparison with before the treatment, *P* < 0.05; ^#^means a comparison with control group, *P* < 0.05.

**Figure 5:** Comparison of the arterial pressure and heart rates in the two groups. (a) The arterial pressure before and at one month after the treatment: The arterial pressure in the two groups at one month after the treatment was significantly lower than it was before the treatment, and the arterial pressure levels in the experimental group were significantly lower than they were in control group (*P* < 0.05). (b) The heart rates before and at one month after the treatment: The heart rates in the two groups after treatment for one month were significantly lower than they were before the treatment, and the heart rates in experimental group were significantly lower than they were in control group (*P* < 0.05). *Note*. ^*∗*^means a comparison with before the treatment, *P* < 0.05; ^#^means a comparison with control group, *P* < 0.05.

**Table 1:** Baseline data of the patients in both groups (*n* = 50).

Classification	Experimental group	Control group	*t*/*X*^2^	*P*
Gender			0.04	0.839
Male	22 (44.00)	21 (42.00)		
Female	28 (56.00)	29 (58.00)		

Age (years old)	67.53 ± 6.44	66.98 ± 7.07	0.42	0.685

BMI (kg/m^2^)	25.12 ± 2.83	24.86 ± 2.49	0.49	0.627

Smoking or not			0.04	0.841
Yes	24 (48.00)	25 (50.00)		
No	26 (52.00)	25 (50.00)		

Drinking or not			0.98	0.545
Yes	23 (46.00)	20 (40.00)		
No	27 (54.00)	30 (60.00)		

Hyperlipidemia			0.04	0.841
Yes	24 (48.00)	23 (46.00)		
No	26 (52.00)	27 (54.00)		

Hypertension			0.36	0.548
Yes	25 (50.00)	22 (44.00)		
No	25 (50.00)	28 (56.00)		

Diabetes mellitus			0.04	0.839
Yes	21 (42.00)	20 (40.00)		
No	29 (58.00)	30 (60.00)		

**Table 2:** Muscle strength grades of the patients in both groups (*n* = 50).

Classification	Experimental group	Control group	*X* ^2^	*P*
0	1	9	7.11	0.008
1	1	10	8.27	0.004
2	1	10	8.27	0.004
3	1	10	8.27	0.004
4	22	5	14.66	<0.001
5	24	6	18.38	<0.001

**Table 3:** Incidence of adverse reactions of the patients in both groups (*n* = 50).

Classification	Experimental group	Control group	*X* ^2^	*P*
Epilepsy (%)	1 (2.00)	5 (10.00)		
Urinary incontinence (%)	1 (2.00)	5 (10.00)		
Pulmonary infection (%)	0 (0.00)	3 (6.00)		
Dementia after stroke (%)	1 (2.00)	2 (4.00)		
Incidence of adverse reactions (%)	3 (6.00)	15 (30.00)	9.76	0.002

**Table 4:** Total effective rate of the patients in both groups (*n* = 50).

Classification	Experimental group	Control group	*X* ^2^	*P*
Markedly effective	25 (50.00)	18 (36.00)	—	—
Effective	21 (38.00)	20 (40.00)	—	—
Ineffective	4 (8.00)	12 (24.00)	—	—
Total effective rate (%)	46 (92.00)	38 (76.00)	4.76	0.03

**Table 5:** Satisfaction of the patients in both groups (*n* = 50).

Classification	Experimental group	Control group	*X* ^2^	*P*
Satisfactory	35 (70.00)	20 (40.00)	—	—
Basic satisfaction	14 (28.00)	15 (30.00)	—	—
Dissatisfaction	1 (2.00)	15 (30.00)	—	—
Satisfaction (%)	49 (98.00)	35 (70.00)	15.48	<0.001

## Data Availability

No data were used to support this study.
